This article has been retracted.

# Effects of Self-Management Intervention Programs Based on the Health Belief Model and Planned Behavior Theory on Self-Management Behavior and Quality of Life in Middle-Aged Stroke Patients

**DOI:** 10.1155/2021/8911143

**Published:** 2021-10-18

**Authors:** Yaoyao Li, Shanshan Zhang, Jie Song, Miao Tuo, Chengmei Sun, Fuguo Yang

**Affiliations:** ^1^School of Nursing, Weifang University of Science and Technology, Weifang, Shandong 262700, China; ^2^General Practice Department, Qingdao Municipal Hospital, Qingdao, Shandong 266071, China; ^3^School of Nursing, Shandong University of Traditional Chinese Medicine, Jinan, Shandong 250355, China; ^4^Neurology Department, Affiliated Hospital of Qingdao University, Qingdao, Shandong 266003, China; ^5^School of Nursing, Qingdao University, Qingdao, Shandong 266071, China

## Abstract

**Objectives:**

To study the effect of self-management intervention programs based on the health belief model and planned behavior theory on self-management behavior and quality of life in middle-aged stroke patients. Most of the intervention studies on the self-management of middle-aged stroke patients focus on traditional Chinese medicine nursing and continuous nursing, lacking theoretical support. In particular, there is a lack of interventions based on the integration of two or more theories.

**Method:**

The middle-aged stroke patients were divided into the control group and the intervention group according to the disease area. A total of 70 patients were included, and 35 patients were included in the control group and the intervention group, respectively. The control group received routine neurological treatment and health education during hospitalization and continued to receive routine health education for 3 months after discharge. On this basis, the intervention group received an intervention program based on an integrated model of health beliefs and planned behavior theory, including 3 health education sessions during hospitalization and 3 months of postdischarge health education. A self-administered stroke general information questionnaire was used to collect basic information on patients' age, gender, and comorbidities. The Stroke Self-Management Behavior Rating Scale and Stroke-Specific Quality-of-Life Scale (SS-QOL) were used to evaluate the management behavior and quality of life of the patients in both groups before and after the intervention.

**Results:**

Before the intervention, there was no statistically significant difference between the two groups in terms of self-management score, quality of life total score, and scores of each dimension (*P* > 0.05). At different periods after the intervention, the total score of self-management, total score of quality of life, and scores of each dimension were significantly higher in both groups than before the intervention (*P* < 0.05). In particular, the self-management and quality of life scores of the intervention group were higher than those of the control group at 1 and 3 months after the intervention (*P* < 0.05).

**Conclusion:**

The self-management intervention scheme based on the integrated model of health belief and planned behavior theory is beneficial to improve the self-management ability and quality of life of stroke patients. It provides basis for clinical nurses to further improve the self-management ability and quality of life of stroke patients. Our findings may also serve as a reference for caregivers in other countries to improve the self-management and quality of life of stroke patients.

## 1. Introduction

Cerebrovascular disease—characterized by high morbidity, mortality, disability, and recurrence rates—is a major cause of disability in the community setting and has become a global public health problem [1–3]. Stroke is a common neurological disease with a continuously rising incidence. In China, every 12 seconds, one person has a stroke [4]. The occurrence and prognosis of cerebral apoplexy bring a heavy blow to the vast majority of patients and their families and also cause a huge loss to the national economy [5].

The incidence of stroke is gradually becoming younger and the trend is global, with data showing that the proportion of stroke patients under 65 years of age is about 30% to 50% of all stroke patients in multiple countries and regions [6–8]. The incidence rate of young and middle-aged stroke patients in China accounts for 10%–14% of the total stroke population [9]. The middle-aged are the important force of the family and the society, bearing the dual responsibility of the family and the society. Once the disease occurs, it is not only a financial burden for the family but also has a significant impact on the society due to the lack of social roles. Therefore, it is particularly important to change the unhealthy behaviors of the middle-aged stroke patients.

Stroke is a behavioral disease. Most stroke patients need to adopt long-term health behaviors to promote disease recovery and improve their health status [10]. In addition, most stroke patients have an acute onset, and long-term effective self-management behaviors are still needed to promote recovery and reduce recurrence rate during convalescence. Self-management behavior refers to patients' self-regulation of physical and mental changes caused by diseases in order to promote their own health, so as to strengthen the management of diseases, diet, medication, daily life, emotions, social activities, and rehabilitation activities [11], which is widely used to improve long-term unhealthy behaviors. Self-management behavior plays an important role in promoting the rehabilitation of stroke patients. Guiding patients to conduct long-term and effective self-management through health education can not only promote the rehabilitation of stroke patients but also improve their daily life ability and quality of life [12, 13]. Therefore, based on health education, it is necessary to provide supportive self-management intervention programs for middle-aged stroke patients.

## 2. Background

At present, most of the intervention studies on the self-management of middle-aged and elderly stroke patients focus on traditional Chinese medicine nursing and continuing nursing, and the self-management intervention can effectively maintain and promote the healthy behavior of stroke patients, change their bad living habits, and improve the prognosis [14, 15]. Studies [16, 17] have shown that health education based on behavioral theory has a higher success rate, and the application of behavioral change theory in relevant studies can strengthen behavioral change and promote the formation of healthy behaviors. The health belief model and the theory of planned behavior are two commonly used theories in the field of health behavior, both of which are widely used in clinical practice. The health belief model includes perceptions of risk, severity, benefits, and barriers and emphasizes the individual's own perceptions and beliefs while ignoring the influence of external pressures such as subjective norms [18]. The theory of planned behavior emphasizes that behavioral attitudes, subjective norms, and perceived behavioral control predict behavioral intentions and behavior but, to some extent, ignores the influence of emotional feelings such as threat and fear on behavior [19, 20]. It follows that a single behavior change theory can only analyze and predict behavior from one perspective, leading to shortcomings in its explanation of behavior.

It has been suggested that combining several different but complementary theories and integrating them to compensate for the shortcomings of a single theory might improve the effectiveness of behavior change theory interventions on behavior [21]. Several researchers have validated the validity of the integrated model of the health belief model and the theory of planned behavior [22]. The results of the study on the behavioral intention of female college students vaccinated with human papillomavirus vaccine showed that the explanatory power of the behavior after the integration of health belief model and planned behavior theory increased [23]. The researchers described the integrated model of health belief model and planned behavior theory but did not discuss the application effect of this model in the self-management of middle-aged stroke patients.

The study aimed to explore the influence of self-management intervention program based on the health belief and planned behavior theory model on the self-management behavior of middle-aged stroke patients, so as to improve the patients' self-management ability, enhance the knowledge of stroke prevention and treatment, and improve their daily activities and quality of life.

## 3. Methods

### 3.1. Design and Sample

Patients were divided into the control group and the intervention group by flipping a coin, among which the subjects enrolled in one ward were the control group and the subjects enrolled in the fourth ward were the intervention group, with 35 cases in each group. The control group received routine neurological treatment and health education during hospitalization and continued to receive routine health education for 3 months after discharge. In addition to the control measures, the intervention group received a self-management intervention based on the integration theory of health beliefs and planned behaviors. The self-management ability and quality of life of the two groups were compared.

The patient was a first-episode stroke patient and was hospitalized in wards 1 and 4 of the Department of Neurology in a general hospital from May to September 2019. Patients to be included in the study must meet the following inclusion criteria: (1) age 45–59 years old; (2) met the diagnostic criteria of the Fourth National Cerebrovascular Disease in 1996, were confirmed by brain CT and MRI, and were all patients with first stroke; (3) with clear consciousness, stable condition, and no communication disorder after treatment; (4) patients or caregivers will use WeChat or other apps; (5) informed consent, voluntary participation in the study. Patients with the following criteria were excluded: (1) with obvious heart, liver, lung, and other organ failure and malignant tumors; (2) a history of mental illness or existing mental disorder; (3) with obvious consciousness disorder and severe cognitive disorder; (4) participating in other research programs. The patient's standard of abscission was (1) unforeseeable circumstances caused by the loss of visitors; (2) voluntarily withdraw from the study; (3) fail to take intervention measures as required; or (4) the disease is not stable, cannot continue to cooperate.

The sample content formula of “comparison of the mean of two samples” was used to estimate the number of samples needed for the study. A total of 70 subjects were included in this study. In the intervention group, 35 cases were studied; 1 case lost contact with the patient, and 1 case withdrew due to the aggravation of the disease during the intervention. In the control group, 35 cases were studied; 1 case withdrew from study due to migration. A total of 67 subjects completed the study, including 33 in the intervention group and 34 in the control group.

### 3.2. Ethical Consideration

This study was approved by the ethics committee of the school and the hospital, and the subjects were informed of the purpose, significance, and methods of this study. After obtaining the consent of the patients, the informed consent was signed.

### 3.3. Interventions

The intervention framework of this study was proposed based on the integrated model of health belief and planned behavior theory, as shown in Figure 1.

#### 3.3.1. Control Group

The control group received routine neurological treatment and health education during hospitalization and continued to receive routine health education for 3 months after discharge. They received hospital health education with the help of neurology nurses, 20–30 minutes each time, including hospital guide (such as detailed introduction to patients on hospital department rules and regulations and the environment, director of the doctors and nurses, reducing anxiety and strangeness, and so on), the matters needing attention of stroke (for example, usually pay attention to exercise and diet low in salt), and discharge guidance. Telephone follow-up was conducted 1 to 3 months after discharge.

#### 3.3.2. Intervention Group

On the basis of the control group, the intervention group received intervention measures based on health beliefs and planned behavior integration theory. The intervention process of the intervention group was divided into two stages: in-hospital health education and postdischarge health education. The intervention mainly includes the following four parts: establishing positive behavior attitude, promoting patients' subjective norms, improving patients' perceived behavior control, and promoting behavioral intention to behavior change. The duration of intervention was during hospitalization and 3 months after discharge. With the support of the head nurse in the department of neurology, the intervention during hospitalization was assisted by the responsible nurse to increase the patient's convincing power. Postdischarge intervention mainly relies on the WeChat group and telephone guidance, and the intervention content was divided into 4 modules and completed within 12 weeks. Health education knowledge was sent to the WeChat group at 20:00 every Friday night, once a week, for 20–30 min each time.

The specific implementation of the intervention was as follows.

- In-hospital health education: during the hospitalization, three face-to-face health education sessions were conducted in the neurology ward, taught by researchers, assisted by the neurology nurse, and attended by patients and their families. The time was 15:00 in the afternoon, 20–30 min each time. The patient was given a self-management manual based on health beliefs and planned behavior theory to clarify the content of self-management intervention, and the patient or family members were invited to join the WeChat group. Assess the patient's disease prevention knowledge, disease management and safe use of drugs, diet, daily life, social life, and motion; through the self-management manual to tell patients with stroke about stroke prevention knowledge, the incidence of stroke, and the influence of stroke onset; let patients know the importance of self-management ability; and improve the patients' sense of crisis. At the same time, patients and their families were informed of the advantages of disease management, diet management, and rehabilitation exercise management, and successful cases of self-management were listed to enhance patients' motivation to change behavior. Finally, the in-hospital health education was organized into words and pictures and sent to the WeChat group to encourage patients and their families to read again and again to help patients establish positive health beliefs.
- Postdischarge health education: health education after discharge was mainly conducted in the form of WeChat group and telephone follow-up, mainly conducted by researchers, with the participation of patients and their families. The time was 20:00 every Friday night, 20–30 min each time.
- 1–2 weeks after discharge (purpose of intervention: to reduce difficulties encountered in self-management): patients were encouraged to speak out about their difficulties in managing themselves. According to the difficulties encountered by the patients in the process of self-management, we will work with the family members to help the patients overcome them. For example, we will demonstrate the rehabilitation actions through videos and pictures until the patients master them. Understood the psychological changes of patients at this stage, mobilized the family members of patients to encourage them to participate in recreational activities, and reduced the impact of negative emotions caused by difficulties in self-management on patients.
- 3–4 weeks after discharge (purpose of intervention: pay attention to the influence of family members and medical workers on patients, improve patients' intention to conduct behavioral change, and promote patients' behavioral change): doctors and rehabilitation therapists in the WeChat group were invited to help explain to patients that self-management management such as disease management and rehabilitation exercise can promote disease recovery and effectively reduce stroke recurrence. The researchers regularly asked the patients about their self-management to make them feel the care of the medical staff and ask their families to accompany them to learn about self-management so that they feel supported from their families.
- 5–8 weeks after discharge (purpose of intervention: to improve the patients' perceptual control ability): according to the investigation of patients' self-management behavior before intervention, the scores of disease management, rehabilitation and exercise, life and living, and diet were lower. Therefore, WeChat group's push content mainly includes the above four aspects: in terms of disease management, the importance of risk factors such as blood pressure and blood glucose was re-emphasized to patients to help them gain confidence in behavioral change; patients were informed of blood pressure and blood glucose measurements and precautions and encouraged to send their measurements to the WeChat group to assist them in establishing behavioral change in disease management. In terms of rehabilitation exercise, the rehabilitation doctor should inform the patients of rehabilitation exercise methods and matters needing attention and send rehabilitation the exercise video to the WeChat group to guide the patients to do simple rehabilitation exercise. In terms of diet, life, and daily life, informing patients about diet and daily life management was the easiest and most effective way to improve patients' confidence in self-management and promote patients' behavior change.
- 9–12 weeks after discharge (purpose of intervention: to improve patients' behavioral intention and promote behavioral intention to behavior shift): the recovered patients or their family members were invited to share their experience and recovery effect in the WeChat group, so as to improve patients' intention of self-management. We summarized feedback every week, praised the progress made by the patients, improved the self-confidence of the patients, and conducted telephone follow-up for patients whose self-management behaviors did not change significantly to find out the reasons, encourage and support the patients, improve the positive emotions of the patients, and enhance the behavioral intention of the patients. Patients were encouraged to share their daily management measures, such as rehabilitation exercise video, in the WeChat group. Researchers corrected the irregular actions in the rehabilitation exercise process of patients, so as to promote the establishment of standardized self-management behaviors of patients. The self-management and stroke prevention knowledge of the patients were regularly questioned in the WeChat group to strengthen the patients' grasp of stroke prevention knowledge.

### 3.4. Evaluation Indicators

In this study, patients' self-management behaviors and intervention effects were evaluated by patients' general information questionnaire, Stroke Self-Management Behavior Rating Scale, and Stroke-Specific Quality-of-Life Scale.

#### 3.4.1. General Information Questionnaire

According to the literature reviewed and the purpose of the study, the researchers designed a questionnaire for the general data of middle-aged stroke patients, which mainly included age, gender, educational level, complications, and other basic information.

#### 3.4.2. Stroke Self-Management Behavior Rating Scale

The Stroke Self-Management Behavior Rating Scale was used to evaluate the stroke self-management behavior, including 7 dimensions, namely disease management, medication management, diet management, daily life and living management, emotion management, social function and interpersonal management, and rehabilitation and exercise management, with a total of 51 items. The Likert 5-point rating scale was used for scoring [24]. Each item was counted as 1–5 points, and the total score of the scale was 51–255 points. The higher the score was, the better the patient's self-management behavior was. Cronbach's coefficient was 0.847 and structure validity was 0.761, indicating that the scale had good content validity and structure validity. This scale is scheduled in patients with cerebral apoplexy in the past 1 month of self-management behavior evaluation; this study's data were collected three times, i.e., for a month after the intervention and 3 months before and after the intervention; the first two data collection time scale content is constant, while the last data collection will be “over the past month” statements in the questionnaire items changed to “over the past three months”.

#### 3.4.3. Stroke-Specific Quality-of-Life Scale

The quality of life of stroke patients was evaluated by the Stroke-Specific Quality-of-Life Scale (SS-QOL) [25]. This scale includes 12 fields: energy, respective family roles, language, activity ability, emotion, personality, self-care ability, social role, thinking, upper limb function, visual acuity, and job/work, each entry evaluated using the Likert 5-point score method, each item 1–5 minutes; the higher the score, the better the patients' health status. Cronbach's coefficient measured by the study was above 0.76 with good validity, and this scale has been widely used to assess the quality of life of stroke patients [26].

### 3.5. Data Collection

The study data were collected three times: once at admission before the intervention and twice after the intervention, i.e., 1 month after the intervention and 3 months after the intervention during telephone follow-up.

### 3.6. Data Analysis

SPSS, version 22.0, was used for data analysis. The measurement data of the intervention group and the control group whose general characteristics were normal distribution were expressed as mean and standard deviation (mean ± SD), while the measurement data of the non-normal distribution were expressed as median (25th percentile, 75th percentile). Enumeration data were represented by frequency and composition ratio (*n*, %). The independent *T*-test, chi-square test, Fisher's exact test, and rank sum test were used to compare the disease-related characteristics. Time effect, intergroup effect, and interaction effect of the control group and intervention group at different time points (baseline, 1 month after intervention, 3 months after intervention) were explained by repeated measures ANOVA. Multivariate analysis of variance (ANOVA) was used to explain differences between groups. For non-normal distribution data with homogeneous variance, a paired sample rank sum test was used to analyze the effects in each group, and two independent sample rank sum tests were used to analyze the differences between groups.

## 4. Results

### 4.1. Demographic Data

Among the 67 subjects, there were 39 males and 28 females. The mean age was (54.40 ± 2.871) years. There were no statistically significant differences in gender and age between the intervention group and the control group (*P* > 0.05) (Table 1).

### 4.2. Results of Outcome Measures

#### 4.2.1. Baseline Comparison of Self-Management Ability Score and Quality of Life Score between the Two Groups

Table 2 shows that there were no statistically significant differences between the two groups in the total score of self-management and scores of all dimensions, total score of quality of life, and scores of all dimensions before intervention (*P* > 0.05).

#### 4.2.2. Comparison of Self-Management Scores between the Two Groups after Intervention

The time effect, intergroup effect, and interaction effect of the self-management total score and the scores of each dimension in the two groups were statistically significant (*P* < 0.001, Table 3). The results of one-way repeated measures analysis of variance showed that the time effect of the self-management total score and the scores of each dimension in the two groups were statistically significant (*P* < 0.001). The total score of self-management and the scores of all dimensions at 3 months after intervention were higher than those at 1 month after intervention and higher than those before intervention, and the difference between the total score of self-management after intervention and the scores of each dimension before intervention was statistically significant (*P* < 0.001). In addition to the rehabilitation and exercise management dimensions of the control group, there were statistically significant differences between the two groups in the total score of self-management and the scores of each dimension 3 months after intervention and 1 month after intervention (*P* < 0.001) (Table 4). Multivariate analysis of variance showed that the total score of self-management and the intergroup effect of the scores of each dimension were statistically significant in the two groups (*P* < 0.001), while the comparison of the total score of self-management and the scores of each dimension before intervention between the two groups showed no statistically significant difference (*P* > 0.05). Compared with the control group, the total score of self-management and scores of all dimensions at 1 month and 3 months after intervention were higher in the intervention group than in the control group, and the difference was statistically significant (*P* < 0.001) (Table 4).

#### 4.2.3. Comparison of Quality of Life Scores between the Two Groups after Intervention

The interaction effects of the total score of quality of life and the scores of each dimension in the two groups were statistically significant (*P* < 0.001, Table 5). Single-factor repetitive measures analysis of variance results show that two groups of the patients' quality of life scores and the time effect of the various dimension scores were statistically significant (*P* < 0.001); the order of the total quality of life scores and the scores of each dimension in the different periods before and after the intervention for the two groups was as follows: 3 months after the intervention > 1 month after the intervention > before the intervention. The differences between the total quality of life scores and the scores of each dimension in different periods after the intervention were statistically significant compared with those before the intervention, and the differences between the total quality of life scores and the scores of each dimension 3 months after the intervention were statistically significant compared with 1 month after the intervention (p<0.001).

Compared with 1 month after intervention, the differences were statistically significant (*P* < 0.001) (Table 6). Multivariate analysis of variance (ANOVA) showed that there were statistically significant effects between the two groups on the total score of quality of life and the scores of each dimension (*P* < 0.001), and there were no statistically significant differences between the two groups on the total score of quality of life and the scores of each dimension before intervention (*P* > 0.05). Compared with the control group, the total score of quality of life and scores of all dimensions at 1 month and 3 months after intervention were higher in the intervention group than in the control group, and the difference was statistically significant (*P* < 0.001) (Table 6).

## 5. Discussion

### 5.1. Intervention Programs Can Improve Patients' Self-Management Ability Based on Health Beliefs and Theory of Planned Behavior

The results of this study showed that the self-management behaviors of patients in the two groups before intervention were at a medium and low level. After the intervention, there were statistically significant differences between the two groups in the total score of self-management and the scores of each dimension before the intervention (*P* < 0.001), and the total score of self-management and the scores of each dimension in the intervention group were higher than those in the control group (*P* < 0.001). It indicates that health education can improve patients' self-management ability, but the intervention model based on health belief and planned behavior integration theory has better effect on improving patients' self-management behavior. Compared with traditional health education, the theoretical basis of this intervention program is an integrated model of health belief model and planned behavior theory. On the one hand, the health belief model solves the problems in the management of stroke, such as the sense of crisis and severity, improves the patients' understanding of stroke, and enhances the attention of middle-aged stroke patients to stroke. Patients are also informed of the benefits of self-management, so as to improve their confidence in self-management and promote their positive behavioral attitude, thus strengthening their intention to conduct behavioral change [27, 28], on the other hand, guided by the theory of planned behavior, giving full play to the perceived behavior control, normative beliefs, and others support for patients to strengthen the patients with the intention of the behavior change and promote the formation of the disease management and rehabilitation of exercise behavior [29, 30]. One month after the intervention, similar results were found for the intervention group with the total score of self-management and scores for each dimension, consistent with existing research, but after 3 months of intervention, the total score of self-management and the scores of all dimensions were higher than those of the intervention group. The intervention model based on the integration theory of health beliefs and planned behaviors and the related continuous nursing can improve patients' self-management behavior, but the nursing model in this study has better effect on improving patients' self-management behavior. The reason for this is that previous studies have only provided continuity of care to patients, without self-management behavioural interventions. In contrast, this study was able to improve patients' self-management and reduce the risk of stroke recurrence by providing behavioural interventions for disease management and rehabilitation exercises under the guidance of health beliefs and the theory of planned behaviour. Studies have shown that intervention schemes with behavioral theory guidance have better intervention effects than those without theoretical guidance [17]. This study applies not only behavioral theory but also two commonly used and complementary theories of behavioral change as the framework, giving full play to the advantages of healthy belief model and planned behavior theory, which greatly improves the intervention effect of this study. However, behavior change is a long-term process, which cannot reflect the intervention effect of self-management in a short time [31]. Therefore, in this study, there was no significant difference in the total score of self-management of patients 1 month after intervention compared with relevant studies. Over time, patients' self-management behaviors were established, and the effect of this study was significantly higher than that of relevant studies [30].

### 5.2. Interventions Can Improve Patients' Quality of Life Based on the Integration of Health Beliefs and Planned Behaviors

There were statistically significant differences between the two groups in the total score of quality of life and the scores of all dimensions before and after the intervention (*P* < 0.001), and the total score of quality of life and the scores of all dimensions in the intervention group were higher than those in the control group (*P* < 0.001). It shows that health education can improve the quality of life of patients, and the intervention model based on the health belief and the integrated theory of planned behavior has a better effect on improving the quality of life of patients. In this study, the patient's quality of life score and each dimension score are higher than those of the related research. To analyse the reasons for this, this study combined subjective criteria, perceived behavioural control and behavioural intention, theory of planned behaviour, and perceived social support to guide patients under the health belief model, and the impact of other control factors on patients was fully considered and acted upon, resulting in greater improvements in quality of life and all dimensions for patients in this study than in previous studies [32]. On the theoretical basis, the theoretical integration model of this study has more advantages. In this study, various interventions were specified, for example, in terms of dietary management, patients were informed that their daily salt intake should not exceed 6 grams, which is about the size of a beer bottle cap. Patients were made aware that better self-management to improve their quality of life was an easy thing to achieve. The patient's family should also be encouraged to improve communication with the patient and to encourage and praise the patient to achieve a higher sense of achievement, creating a virtuous circle. Therefore, the total score of quality of life in the intervention group was higher than that in the control group. In this study, the intervention group after the intervention of family roles scores higher than that of related research [33]; previous studies have ignored the family factors such as the influence on patients; and under the guidance of theory of integration model, this study combined with preintervention survey, considering the midlife stroke patient's stage of life, gives full play to the role of the medical personnel, family, and other social support. Encourage patients to communicate with their families, medical staff, and patients, and assist patients to adjust their mentality as soon as possible to complete the transformation of family role.

## 6. Conclusion

Self-management intervention scheme based on health belief and integrative theory of planned behavior is beneficial to improve the self-management ability of middle-aged stroke patients and promote their adoption of healthy behaviors. It is beneficial to improve the knowledge level of prevention and treatment of stroke in middle-aged and elderly patients and enhance the understanding of stroke disease, promote the daily life ability of the middle-aged stroke patients, and enhance their confidence to return to the family and society, so as to improve the quality of life of middle-aged stroke patients.

### 6.1. Limitations of the Study

Because the researchers' time, resources, and energy into the research object of this study are limited to a level of first-class comprehensive hospitals, many hospitals and community hospitals in other areas are not included in the intervention of the present study time and follow-up for 3 months, and since the time is limited, based on the health belief and the consolidation theory of planned behavior intervention model, long-term outcomes in patients with cerebral apoplexy in middle age have not yet been verified. The emotional aspects of stroke were not assessed in this study. It is suggested that future studies should expand the evaluation of cerebral pain emotion and further explore the effect of this intervention mode.

### 6.2. Relevance to Practice

This study applied an intervention programme based on an integrated model of health beliefs and behaviours to middle-aged stroke patients. It improved middle-aged stroke patients' self-management skills, stroke prevention knowledge, daily activity skills, quality of life, and self-care skills.

## Figures and Tables

**Figure 1:** Block diagram of self-management intervention.

**Table 1:** Demographic data of subjects in the groups.

	Total object of study (*n* = 67)	Intervention group (*n* = 33)	Control group (*n* = 34)	Statistics	*P*
Age (mean ± SD, years)	54.40 ± 2.87	54.36 ± 3.30	54.44 ± 2.44	−0.110^a^	0.913
*Gender (n, %)*					
Male	39(58.20)	23(69.70)	16(47.10)	3.528^b^	0.084
Female	28(41.80)	10(30.30)	18(52.90)		

*Education (n, %)*					
≤Middle school	35(52.20)	15(45.50)	20(58.80)	−0.488^c^	0.677
High school	24(35.80)	16(48.50)	8(23.50)		
≥College	8(12.00)	2(6.00)	6(17.70)		

*Marital status (n, %)*					
Married	63(94.00)	32(97.00)	31(91.20)	1.871^d^	0.742
Divorced or separated	2(3.00)	0(0.00)	2(5.90)		
Death of a spouse	2(3.00)	1(3.00)	1(2.90)		

*Status of children (person) (n, %)*					
1	6(9.00)	2(6.10)	4(11.80)	−0.811^c^	0.673
≥2	61(91.00)	31(93.90)	30(88.20)		

*Professional (n, %)*					
Farmers	15(22.40)	5(15.20)	10(29.30)	4.083^d^	0.417
Workers	27(40.30)	15(45.50)	12(35.30)		
Cadres	7(10.40)	3(9.10)	4(11.80)		
Soho	12(17.90)	8(24.20)	4(11.80)		
Other	6(9.00)	2(6.00)	4(11.80)		

*Monthly per capita household income (n, %)*					
<1000 yuan	1(1.50)	1(3.00)	0	−0.130^c^	0.892
1000～5000 yuan	49(73.10)	23(69.70)	26(76.50)		
>5000 yuan	17(25.40)	9(27.30)	8(23.50)		

*Medical payment method (n, %)*					
Medical insurance	40(59.70)	19(57.60)	21(61.80)	1.042^d^	0.899
New rural cooperative medical care	26(38.80)	13(39.40)	13(38.20)		
Own expense	1(150)	1(3.00)	0(0.00)		

*Combined with other diseases (n, %)*					
0	9(13.40)	5(15.20)	4(11.80)	−0.017^c^	0.923
1	51(76.10)	24(72.70)	27(79.40)		
≥2	7(10.50)	4(12.10)	3(8.80)		

*Access to disease knowledge (n, %)*					
Television and radio	46(68.70)	24(72.70)	22(64.70)	3.534^d^	0.699
Lectures and related activities	3(4.50)	1(3.10)	2(5.90)		
Medical staff	5(7.50)	3(9.10)	2(5.90)		
Books	1(1.50)	0(0.00)	1(2.90)		
Other stroke patients	5(7.50)	1(3.10)	4(11.80)		
Caregivers	7(10.30)	4(12.00)	3(8.80)		
Other	0 (0.00)	0(0.00)	0(0.00)		

*Stroke type (n, %)*					
Hemorrhagic stroke	8(11.90)	5(15.20)	3(8.80)	0.638^b^	0.476
Ischemic stroke	59(88.10)	28(84.80)	31(91.20)		

*Smoking (n, %)*					
Yes	15(22.40)	8(24.20)	7(20.60)	0.129^b^	0.776
No	52(77.60)	25(75.80)	27(79.40)		

Note: ^a^*T*-test; ^b^chi-square test; ^c^rank sum test; ^d^Fisher's exact probability.

**Table 2:** The two groups of patients before the intervention of self-management behavior, quality of life total score, and each dimension score (mean ± SD, scores).

	Intervention group (*n* = 33)	Control group (*n* = 34)	*t*	*P*
Total score of self-management	117.09 ± 4.25	117.06 ± 3.37	0.034	0.973
Disease management	15.70 ± 1.70	15.76 ± 1.58	−0.169	0.866
Management of safe drug use	13.82 ± 1.99	13.85 ± 1.56	−0.08	0.937
Dietary management	21.42 ± 1.92	21.50 ± 1.97	−0.159	0.874
Life management	21.88 ± 2.18	21.41 ± 1.88	0.942	0.350
Emotion management	17.33 ± 1.41	17.32 ± 1.49	0.028	0.978
Social management	13.45 ± 2.56	13.47 ± 1.60	−0.031	0.975
Rehabilitation exercise management	13.48 ± 1.72	13.74 ± 1.42	−0.651	0.517
Total score of quality of life	135.55 ± 3.93	135.56 ± 4.52	−0.013	0.990
Energy	7.21 ± 1.14	7.35 ± 1.10	−0.515	0.608
Family roles	6.85 ± 0.87	7.06 ± 0.81	−1.022	0.311
Language	13.85 ± 1.52	13.88 ± 1.43	−0.094	0.926
Activity ability	17.12 ± 1.27	17.24 ± 1.42	−0.347	0.730
Emotion	14.30 ± 1.55	14.18 ± 1.31	0.361	0.719
Personality	7.85 ± 1.37	8.03 ± 1.27	−0.561	0.577
Self-care ability	15.61 ± 1.48	15.35 ± 1.59	0.674	0.503
Social role	14.15 ± 1.52	14.18 ± 1.57	−0.066	0.948
Thinking	7.33 ± 0.99	7.35 ± 1.20	−0.073	0.942
Upper limb function	12.36 ± 1.41	12.50 ± 1.26	−0.417	0.678
Vision	10.06 ± 0.66	9.71 ± 0.91	1.829	0.072
Work	8.85 ± 1.09	8.74 ± 1.05	0.432	0.667

**Table 3:** Results of self-management and repeated measures ANCOVA at 3 time points in two groups.

	Time effect		Intergroup effect		The interaction effect	
	*F*	*P*	*F*	*P*	*F*	*P*
Total score of self-management	4450.631	<0.001	1551.058	<0.001	1000.379	<0.001
Disease management	2481.479	<0.001	530.840	<0.001	532.644	<0.001
Management of safe drug use	643.547	<0.001	139.788	<0.001	88.342	<0.001
Dietary management	631.522	<0.001	226.957	<0.001	172.207	<0.001
Life management	541.755	<0.001	589.507	<0.001	145.705	<0.001
Emotion management	418.369	<0.001	42.792	<0.001	20.575	<0.001
Social management	700.490	<0.001	210.147	<0.001	98.969	<0.001
Rehabilitation exercise management	463.976	<0.001	614.199	<0.001	248.432	<0.001

**Table 4:** Self-management and scores of each dimension were compared between the two groups (mean ± SD, scores).

		n	Before the intervention	After the intervention		*F*	*P*
				1 month	3 months		
Total score of self-management	Intervention group	33	117.09 ± 4.25	189.39 ± 6.30^a^	221.36 ± 3.27^ab^	4127.470	0.016
	Control group	34	117.06 ± 3.37	141.59 ± 7.91^a^	154.65 ± 5.54^ab^	355.110	＜0.001
	*t*		0.032	27.309	59.791		
	*P*		0.975	<0.001	<0.001		

Disease management	Intervention group	33	15.70 ± 1.70	33.36 ± 3.01^a^	42.82 ± 2.38^ab^	1064.930	<0.001
	Control group	34	15.76 ± 1.58	23.00 ± 1.46^a^	25.56 ± 1.86^ab^	325.830	<0.001
	*t*		0.150	18.008	33.131		
	*P*		0.882	<0.001	<0.001		

Management of safe drug use	Intervention group	33	13.82 ± 1.99	22.18 ± 1.24^a^	23.82 ± 0.58^ab^	488.090	<0.001
	Control group	34	13.85 ± 1.56	17.12 ± 1.70^a^	18.85 ± 1.79^ab^	77.120	<0.001
	*t*		0.069	13.884	15.192		
	*P*		0.945	<0.001	<0.001		

Dietary management	Intervention group	33	21.42 ± 1.92	30.33 ± 2.27^a^	35.03 ± 1.74^ab^	398.650	<0.001
	Control group	34	21.50 ± 1.97	23.03 ± 1.36^a^	26.15 ± 2.02^ab^	58.390	<0.001
	*t*		0.168	16.023	19.254		
	*P*		0.867	<0.001	<0.001		

Life management	Intervention group	33	21.88 ± 2.18	33.09 ± 1.81^a^	37.45 ± 1.09^ab^	693.000	<0.001
	Control group	34	21.41 ± 1.88	24.06 ± 2.64^a^	26.71 ± 1.40^ab^	57.470	<0.001
	*t*		0.989	16.281	34.965		
	*P*		0.327	<0.001	<0.001		

Emotion management	Intervention group	33	17.33 ± 1.41	20.48 ± 1.33^a^	23.79 ± 0.78^ab^	236.650	<0.001
	Control group	34	17.32 ± 1.49	18.91 ± 1.11^a^	21.47 ± 0.83^ab^	107.980	<0.001
	*t*		0.028	5.252	11.782		
	*P*		0.978	<0.001	<0.001		

Social management	Intervention group	33	13.45 ± 2.56	24.03 ± 1.63^a^	28.00 ± 1.30^ab^	513.750	＜0.001
	Control group	34	13.47 ± 1.60	18.47 ± 2.26^a^	20.00 ± 1.61^ab^	115.960	＜0.001
	*t*		0.038	11.520	22.337		
	*P*		0.970	<0.001	<0.001		

Rehabilitation exercise management	Intervention group	33	13.48 ± 1.72	25.91 ± 2.24^a^	30.45 ± 1.79^ab^	683.46	<0.001
	Control group	34	13.74 ± 1.42	17.00 ± 2.03^a^	15.91 ± 2.73^a^	20.670	<0.001
	*t*		0.676	17.070	25.698		
	*P*		0.502	<0.001	<0.001		

Note: ^a^comparison with preintervention (*P* < 0.001); ^b^compared with 1 month after the intervention (*P* < 0.001).

**Table 5:** Results of repeated measures ANCOVA of quality of life and scores of each dimension at 3 time points in two groups.

	Time effect		Intergroup effect		The interaction effect	
	*F*	*P*	*F*	*F*	*P*	*F*
Total score of quality of life	15912.903	<0.001	417.515	<0.001	856.822	<0.001
Energy	1008.836	<0.001	37.816	<0.001	46.885	<0.001
Family roles	1030.537	<0.001	85.723	<0.001	63.618	<0.001
Language	1203.099	<0.001	48.601	<0.001	81.684	<0.001
Activity ability	1373.207	<0.001	99.989	<0.001	81.870	<0.001
Emotion	985.334	<0.001	56.716	<0.001	48.674	<0.001
Personality	544.274	<0.001	40.822	<0.001	35.779	<0.001
Self-care ability	836.941	<0.001	69.700	<0.001	43.550	<0.001
Social role	1102.515	<0.001	46.799	<0.001	58.014	<0.001
Thinking	1095.500	<0.001	42.926	<0.001	53.806	<0.001
Upper limb function	1711.449	<0.001	76.254	<0.001	99.727	<0.001
Vision	719.166	<0.001	59.364	<0.001	29.928	<0.001
Work	863.835	<0.001	35.097	<0.001	36.512	<0.001

**Table 6:** The quality of life and scores of each dimension were compared between the two groups (mean ± SD, scores).

		*n*	Before the intervention	After the intervention		*F*	*P*
				1 month	3 months		
Total score of quality of life	Intervention group	33	135.55 ± 3.93	192.03 ± 5.64^a^	227.21 ± 3.77^ab^	3605.010	<0.001
	Control group	34	135.56 ± 4.52	162.50 ± 4.53^a^	195.74 ± 4.63^ab^	1485.680	<0.001
	*t*		0.010	23.664	30.456		
	*P*		0.992	<0.001	<0.001		

Energy	Intervention group	33	7.21 ± 1.14	11.00 ± 0.71^a^	13.73 ± 0.88^ab^	411.700	<0.001
	Control group	34	7.35 ± 1.10	9.50 ± 0.99^a^	11.62 ± 0.85^ab^	159.630	<0.001
	*t*		0.512	7.108	9.983		
	*P*		0.612	<0.001	<0.001		

Family roles	Intervention group	33	6.85 ± 0.87	11.00 ± 0.97^a^	13.76 ± 0.97^ab^	453.897	<0.001
	Control group	34	7.06 ± 0.81	9.00 ± 0.65^a^	11.38 ± 0.78^ab^	283.070	<0.001
	*t*		1.023	9.942	11.084		
	*P*		0.310	<0.001	<0.001		

Language	Intervention group	33	13.85 ± 1.52	18.91 ± 1.83^a^	23.21 ± 1.05^ab^	134.050	<0.001
	Control group	34	13.88 ± 1.43	16.12 ± 1.45^a^	19.50 ± 1.35^ab^	136.760	<0.001
	*t*		0.083	6.928	12.530		
	*P*		0.934	<0.001	<0.001		

Activity ability	Intervention group	33	17.12 ± 1.27	24.70 ± 1.76^a^	28.30 ± 1.02^ab^	560.650	<0.001
	Control group	34	17.24 ± 1.42	20.79 ± 1.18^a^	24.56 ± 1.21^ab^	280.480	<0.001
	*t*		0.364	10.710	13.659		
	*P*		0.718	<0.001	<0.001		

Emotion	Intervention group	33	14.30 ± 1.55	18.58 ± 1.39^a^	23.27 ± 1.13^ab^	355.130	<0.001
	Control group	34	14.18 ± 1.31	16.00 ± 1.33^a^	20.00 ± 1.30^ab^	174.710	<0.001
	*t*		0.343	7.764	11.166		
	*P*		0.733	<0.001	<0.001		

Personality	Intervention group	33	7.85 ± 1.37	12.39 ± 1.30^a^	14.03 ± 0.73^ab^	249.470	<0.001
	Control group	34	8.03 ± 1.27	10.18 ± 1.19^a^	12.03 ± 0.80^ab^	111.410	<0.001
	*t*		0.558	7.262	10.680		
	*P*		0.579	<0.001	<0.001		

Self-care ability	Intervention group	33	15.61 ± 1.48	21.06 ± 1.35^a^	23.76 ± 0.90^ab^	353.800	<0.001
	Control group	34	15.35 ± 1.59	17.94 ± 1.23^a^	20.94 ± 1.04^ab^	155.830	<0.001
	*t*		0.213	9.894	11.853		
	*P*		0.832	<0.001	<0.001		

Social role	Intervention group	33	14.15 ± 1.52	19.27 ± 1.28^a^	23.03 ± 1.10^ab^	381.270	<0.001
	Control group	34	14.18 ± 1.57	16.59 ± 1.42^a^	19.97 ± 1.19^ab^	146.310	<0.001
	*t*		0.079	8.106	10.921		
	*P*		0.937	<0.001	<0.001		

Thinking	Intervention group	33	7.33 ± 0.99	11.52 ± 0.80^a^	13.55 ± 0.97^ab^	388.920	<0.001
	Control group	34	7.35 ± 1.20	9.41 ± 0.93^a^	11.65 ± 0.98^ab^	144.480	<0.001
	*t*		0.074	9.943	7.974		
	*P*		0.941	<0.001	<0.001		

Upper limb function	Intervention group	33	12.36 ± 1.41	18.97 ± 0.95^a^	22.24 ± 1.09^ab^	614.900	<0.001
	Control group	34	12.50 ± 1.26	15.44 ± 1.33^a^	19.15 ± 1.18^ab^	238.520	<0.001
	*t*		0.429	12.468	11.125		
	*P*		0.670	<0.001	<0.001		

Vision	Intervention group	33	10.06 ± 0.66	13.15 ± 1.09^a^	14.42 ± 0.61^ab^	250.360	<0.001
	Control group	34	9.71 ± 0.91	11.38 ± 0.78^a^	12.82 ± 0.72^ab^	54.730	<0.001
	*t*		1.798	7.662	9.800		
	*P*		0.077	<0.001	<0.001		

Work	Intervention group	33	8.85 ± 1.09	11.48 ± 0.76^a^	13.91 ± 0.91^ab^	244.440	<0.001
	Control group	34	8.74 ± 1.05	10.15 ± 0.74^a^	12.12 ± 0.69^ab^	138.27	<0.001
	*t*		0.421	7.258	9.090		
	*P*		0.675	<0.001	<0.001		

Note: ^a^comparison with preintervention (*P* < 0.001); ^b^compared with 1 month after the intervention (*P* < 0.001).

## Data Availability

The primary data to support the results of this study are available upon reasonable request to the corresponding author.
